# Early Diagnosis of Brain Tumour MRI Images Using Hybrid Techniques between Deep and Machine Learning

**DOI:** 10.1155/2022/8330833

**Published:** 2022-05-18

**Authors:** Ebrahim Mohammed Senan, Mukti E. Jadhav, Taha H. Rassem, Abdulaziz Salamah Aljaloud, Badiea Abdulkarem Mohammed, Zeyad Ghaleb Al-Mekhlafi

**Affiliations:** ^1^Department of Computer Science, Hajjah University, Hajjah, Yemen; ^2^Shri Shivaji Science & Arts College, Chikhli Dist., Buldana, India; ^3^Faculty of Science and Technology, Bournemouth University, Poole, UK; ^4^College of Computer Science and Engineering, University of Hail, Hail, Saudi Arabia

## Abstract

Cancer is considered one of the most aggressive and destructive diseases that shortens the average lives of patients. Misdiagnosed brain tumours lead to false medical intervention, which reduces patients' chance of survival. Accurate early medical diagnoses of brain tumour are an essential point for starting treatment plans that improve the survival of patients with brain tumours. Computer-aided diagnostic systems have provided consecutive successes for helping medical doctors make accurate diagnoses and have conducted positive strides in the field of deep and machine learning. Deep convolutional layers extract strong distinguishing features from the regions of interest compared with those extracted using traditional methods. In this study, different experiments are performed for brain tumour diagnosis by combining deep learning and traditional machine learning techniques. AlexNet and ResNet-18 are used with the support vector machine (SVM) algorithm for brain tumour classification and diagnosis. Brain tumour magnetic resonance imaging (MRI) images are enhanced using the average filter technique. Then, deep learning techniques are applied to extract robust and important deep features via deep convolutional layers. The process of combining deep and machine learning techniques starts, where features are extracted using deep learning techniques, namely, AlexNet and ResNet-18. These features are then classified using SoftMax and SVM. The MRI dataset contains 3,060 images divided into four classes, which are three tumours and one normal. All systems have achieved superior results. Specifically, the AlexNet+SVM hybrid technique exhibits the best performance, with 95.10% accuracy, 95.25% sensitivity, and 98.50% specificity.

## 1. Introduction

Cancer is one of the biggest health problems and challenges that threatens the life of humanity nowadays. After cardiovascular disorders, cancer is the second leading cause of death [1], where every sixth death is due to cancer. Among the different types of cancer, brain tumours are the most dangerous and deadly due to their heterogeneous characteristics, aggressive nature, and low survival rate. Brain tumours have numerous forms based on their shape, texture, and location, such as meningioma, glioma, acoustic neuroma, pituitary, and lymphoma [2]. The incidence of brain tumours is about 45%, 15%, and 15% for glioma, meningioma, and pituitary tumours, respectively [3]. Diagnosis is made depending on the tumour type and location, so doctors can predict patients' survival and make decisions about treatments that range from surgery to chemotherapy and radiotherapy. Therefore, a proper diagnosis of the tumour type is important in planning treatments and monitoring patients' conditions [4]. Magnetic resonance imaging (MRI) is a medical imaging technique that produces clear images of the body's internal organs without causing pain or requiring surgery, in 2D and 3D formats. It is one of the most widely used high-precision techniques for cancer detection and diagnosis [5]. However, identifying the tumour type through MRI is time-consuming, difficult, and error-prone, thereby requiring highly experienced radiologists. Due to the tumour diversity, visible features in MRI images, which enable proper decision-making, sometimes do not exist. Therefore, humans cannot easily rely on manual diagnoses. Moreover, the underdiagnosis of brain tumours is dangerous, as it reduces the response to treatments and the survival rate. Correct diagnoses help patients receive accurate treatments and survive for a long time. Accordingly, the need to use artificial intelligence (AI) techniques has become essential in diagnosing medical images, such as MRI images by the computer-aided diagnosis (CAD) system [6]. Such techniques are used to reduce workload and assist doctors and radiologists in making accurate diagnoses [7]. The CAD system comprises several stages, such as the preprocessing phase where noise is removed from images [8]; the segmentation stage where the lesion area is identified and isolated from the rest of the images [9]; the feature extraction stage where the most important features, which represent the tumour, are extracted [8]; and the classification stage where each image is classified and abnormality is predicted [10]. The literature review reveals that many machine learning algorithms have been used to classify MRI images [11–13]. Many deep learning techniques are recently used for diagnosing MRI images [14–16], which are parts of machine learning that do not require manual features. In this study, we analyse and evaluate the performance of AlexNet and ResNet-18 deep learning models for the early diagnosis of brain tumours. To evaluate the performance of deep learning (AlexNet and ResNet-18) and machine learning (support vector machine (SVM)) techniques, they are called AlexNet+SVM and ResNet-18+SVM for the early detection of brain tumours from MRI images.

The main contributions of this paper are as follows:

- Hybrid deep and machine learning techniques are applied where images are optimised to remove noise before they are introduced into deep learning techniques for extracting the most important deep discriminatory features; classification algorithms for convolutional neural networks (CNNs) through SoftMax and machine learning through the SVM algorithm are applied
- Different structures of the CNNs of two AlexNet and ResNet-18 models and their deployment are explored to classify the MRI images of brain tumours by using a learning transfer technique
- The proposed models preserve the most important local distinguishing features through the hypercolumn technique, which provides features that are inherent in the previous layer, for transfer to the next layer to increase the classification performance
- The proposed models also present a promising and high-sensitivity diagnostic model for diagnosing MRI images to classify brain tumours and support the decisions of experts and radiologists

The rest of this paper is organised as follows: Section 2 reviews relevant previous studies.  Section 3 provides an overview of deep and machine learning networks.  Section 4 introduces the materials and methods for analysing MRI images.  Section 5 presents the detailed explanations of the classification methods using CNNs and hybrid methods.  Section 6 provides the experiment results.  Section 7 discusses and compares the results with relevant studies. Section 8 concludes the paper.

## 2. Related Work

In this section, we present a group of previous studies related to the diagnosis of brain tumours. However, many researchers dedicate their efforts to reach promising results in diagnosing brain tumours. In this study, several techniques have been applied that have yielded promising results in diagnosing brain tumours.

Narmatha et al. proposed a fuzzy brainstorm optimisation different method to classify MRI images for a brain tumour dataset. This technique is a combination of fuzzy and brainstorm optimisation techniques. Brainstorm optimisation puts on-cluster centers on focus and gives them the highest priority, whereas fuzzy builds on multiple iterations to provide an optimal network structure. They used the brain tumour segmentation (BraTS) 2018 dataset, and their proposed system reached 93.85% accuracy, 95.77% sensitivity, 94.77% precision, and 95.42% *F*1 score [17]. Sharif et al. have proposed a different methodology for active deep learning-based feature selection for brain tumour segmentation and classification. Contrast enhancement was applied for the saliency map construction, which applies the threshold to convert to binary. The InceptionV3 pretrained model was also applied to extract deep features, which are combined with the dominant rotated LBP features for improved texture analysis. Then, particle swarm optimisation (PSO) was conducted to optimise the concatenated vectors and classify them using the SoftMax function. The authors used two datasets, BraTS 2017 and BraTS 2018. With the BraTS 2017 dataset, the system achieved dice scores of 83.73%, 93.7%, and 79.94% for a core tumour, a whole tumour, and an enhanced tumour, respectively. With the BraTS 2018 dataset, the system yielded dice scores of 88.34%, 91.2%, and 81.84% for a core tumour, a whole tumour and an enhanced tumour, respectively [18], while Dandu et al. detected brain and pancreatic tumours by using a new technique called the decision-based couple window median filter (DBCWMF) algorithm, cat swarm optimisation (CSO), statistical region merging (SRM), and scale-invariant feature transform (SIFT). CSO–SIFT extraction and backpropagation neural network (BPNN) classification algorithms were also used. The DBCWMF algorithm optimised images, whereas the SRM algorithm segmented images and identified lesion areas. CSO and SIFT techniques were used to extract features from lesion areas. The BPNN algorithm was employed to classify tumours. A dataset from the Harvard Medical School and the Cancer Imaging Archive database was used in their experiments. The system achieved an accuracy of 90.2% [19]. While Amin et al. proposed a process of combining the texture and structural features of four MRI image sequences, namely, T1C, T1, Flair, and T2, to detect brain tumours, the fusion process was carried out by a discrete wavelet transform along with Daubechies wavelet kernel. Subsequently, they applied a partial differential diffusion filter to remove unwanted artifacts. Next, a global thresholding algorithm was used to segment lesion areas. The performance of the proposed system was evaluated on five BraTS datasets. The results using fused images were better than those using individual sequences in the dataset. The methodology achieved an accuracy of 87%, a sensitivity of 92%, and a specificity of 80% [20]. Huang et al. presented a new method based on complex networks (CNNBCN) and modified the activation function for diagnosing the MRI images of brain tumours. Randomly generated graph algorithms provided the network structure. A network generator mapped these graphs into a computable network. Their proposed CNNBCN system reached 94.53% accuracy. Although CNN models achieved better results than their CNNBCN method in diagnosing brain tumours, their method enriches CNN design [21]. Kaur et al. implemented several pretrained deep convolutional neural networks (DCNNs), namely, AlexNet, GoogLeNet, ResNet101, ResNet50, VGG16, InceptionV3, and InceptionResNetV2, where they replaced the last layers of these models to suit the new classes of images. These models were evaluated on a dataset from the benchmark Figshare repository, Harvard, and clinics. The dataset was divided into 60% for training and 40% for testing. All their experiences proved that the AlexNet model achieves the best performance in less time than other models. The method reached an accuracy of 91.51%, a sensitivity of 90.65%, and a specificity of 95.79% with the Figshare repository dataset [22]. Raja et al. developed a novel system that differs from the literature for classifying brain tumours by using a hybrid deep autoencoder (DAE) with a Bayesian fuzzy clustering- (BFC-) based segmentation algorithm. They applied a nonlocal mean filter to remove noise and distortion. Subsequently, they applied the BFC algorithm to segment the tumour region. Then, robust features were extracted using methods such as scattering transform, information-theoretic measures, and wavelet packet Tsallis entropy. Finally, they applied a hybrid scheme of the DAE-based Jaya optimisation algorithm to classify brain tumours. The system performance was evaluated on the BraTS 2015 dataset. Their system achieved 98.5% accuracy [23]. Kumar et al. presented a novel stationery, wavelet-based radiomics approach for a highly accurate noninvasive classification of glioma. The system performance was evaluated on the BraTS dataset, and the calculation was performed according to the radiomics features of three interesting regions. These characteristics were classified using the random forest algorithm; the proposed system reached 97.54% accuracy, 97.62% sensitivity, and 97.33% specificity [24]. Bhanothu et al. presented an R-CNN model for brain tumour detection and tumour region selection using the Region Proposal Network (RPN). The proposed method uses the VGG-16 model structure as the primary seed for tumour differentiation and classification. The system achieved an average precision of 77.60% [25]. Kumar et al. presented a new method called Dolphin-SCA based on deep learning models to diagnose brain images and improve accuracy. MRI images were enhanced, and tumour area segmentation was done by fuzzy deformable fusion based on the Dolphin Sine Cosine method. Then, the features were extracted according to the power LDP, statistical features, and DCNNs. System performance was evaluated on BraTS and SimBraTS databases, achieving 96.3% accuracy [26]. Muhammed et al. presented a methodology for the diagnosis of brain tumours. The methodology consists of several steps: using an edge-based histogram equalisation to show linear variance and discrete cosine transform. Extract deep feature maps by VGG16 and VGG19 models. Then, select the best features using an extreme learning machine (ELM) and combine the variable features into a single matrix using a partial less square; finally, fed feature matrix to ELM for diagnosis. The method achieved an accuracy of 92.5% with the BraTs2018 dataset [27]. Raheleh et al. (2020) designed a hybrid model for classifying images in a brain tumour dataset; firstly, all images were optimised to remove noise. Secondly, the dataset was trained on a hybrid model between CNN and neural autoregressive distribution estimation. The hybrid model yielded good results for diagnosing the brain tumour dataset, as the hybrid model reached an accuracy of 89.8% for diagnosing meningioma, 95.2% for glioma, and 98.5% for pituitary tumour [28]. Muhmmad et al. (2020) applied a different approach to select active features based on CNN models for tumour region segmentation and diagnosis. Image contrast was improved, and a saliency map was constructed and converted to a 2D format. Features were extracted using the local binary pattern algorithm and combined with deep feature maps. PSO was also implemented to improve the features of the sequenced vector. The methodology achieved segmentation on the dataset with a dice score of 83.73% for the primary tumour and the whole tumour with a score of 93.7% [18]. Wentao et al. (2020) suggested a different methodology for preserving information during the encoding and decoding processes. The methodology involves integrating DCNNs with SVM. It goes through three stages: firstly, CNNs are trained to map only the tumour area. Secondly, all the classes in CNNs are named, and the networks are trained by using SVM. Thirdly, deep classifier training was performed by integrating CNNs with SVM. The methodology reached a DSC of 89.58% and a sensitivity of 91.10% for diagnosing brain tumours [29]. Muhammad et al. (2020) proposed a new methodology that is based on statistical advantages to classify them using machine learning algorithms. All images were enhanced with a median filter to remove noise and were converted from greyscale to RGB. Colour features were extracted from each image and categorised by an artificial neural network (ANN), naïve Bayes, *k*-nearest neighbour network (KNN), and decision tree algorithms. The decision tree algorithm achieved the best results among other classifiers. The method achieved an *F*1 score of 83%, recall of 83%, and precision of 85% [30].

## 3. Overview

### 3.1. Deep Learning

Deep neural network learning techniques have been introduced to improve the performance of accurate diagnoses of various medical images and to assist doctors and radiologists in diagnosing diseases in their early stages. Medical images contain complex sizes, shapes, and colours that are difficult for CNNs to directly train. The curriculum learning strategy is used to solve this complex problem, which includes gradual training to solve complex concepts. To improve CNN performance and reduce overfitting, deep learning techniques require large amounts of data. However, obtaining large datasets for serious medical diseases is difficult. Thus, CNNs perform augmentation to overcome this problem. CNNs comprise convolutional, pooling, and fully connected layers. Convolutional layers extract features by specifying patterns, lines, edges, shapes, and colours. These layers convolve the input array with convolution kernels in each hidden layer of CNN. Multiple kernels produce multiple and deep features that are successful in vision tasks, such as classification. Between these convolutional layers are feature maps called pooling layers that collect features locally and spatially. The basic task of pooling layers is the maximum or average value transfers and thus reduces feature dimensions (reducing the feature map size). The DCNN architecture comprises convolutional and pooling layers, which operate repeatedly. At the end of CNNs, the architecture comprises fully connected layers attached to the classification and regression tasks that lead to the final decision-making. During the training phase, the loss is estimated by comparing actual and predicted values [31]. Given that the CNN architecture consists of several layers, the training data reach millions of parameters. That is, DCNNs require thousands of images to reach promising classification accuracy. Thus, CNNs provide data augmentation techniques by transformation methods, such as scaling, rotation, flipping, and translation. In this study, two models of CNN technologies are used, namely, AlexNet and ResNet-18 [32].

### 3.2. Machine Learning

Machine learning is the ability to learn by training data and adapt to solve future problems without human intervention. Machine learning models fine-tune training data to produce accurate predictions. The main goal of modules is their ability to generalise their acquired experience and to make accurate predictions of the test data. Generalisation is tuned during the training phase using a training dataset, and a validation set is used to adjust model parameters. After several iterations of the training and validation phases, the model performance is tested on the test set. Many machine learning algorithms exist, namely, SVM, KNNs, ANNs [33], feed-forward neural networks [34], and BPNNs [35], all of which have proven their superior ability to classify biomedical images, such as the MRI images of brain tumours.

## 4. Materials and Methods

Many experiments are performed to evaluate AlexNet and ResNet and after their integration with SVM for brain tumour detection. The general structure of the brain tumour detection system used in this study is shown in Figure 1. In the preprocessing stage, the average filter is used to remove noise. This filter smoothens images by reducing the contrast among adjacent pixels. All feature images are extracted through convolutional layers where AlexNet and ResNet-18 models are applied to extract the shape, colour, and texture features of brain tumours through convolutional layers. A total of 9,216 features are extracted for each MRI image. Thus, the feature map size is 3060 (image) × 9216 (feature). All images are also diagnosed using deep learning techniques for two models, namely, AlexNet and ResNet-18, through SoftMax and by using machine learning techniques through SVM. The performance of each classifier is evaluated using measures of accuracy, sensitivity, and specificity.

AlexNet and ResNet-18 architectures are mentioned. Their overall architecture comprises convolutional, pooling, and fully connected layers. Convolutional layers work by wrapping filters (3 × 3 and 5 × 5) on each input image and extracting local distinguishing features. These features are transferred to the next layer. Features are preserved in activation maps, which determine the most efficient features. Pooling layers reduce the size of the input image and speed up the process by reducing the image dimensions and minimising the architecture cost. Fully connected layers determine the most effective features and transfer them to the classification layers, which perform the classification process according to the number of classes. In this study, deep and machine learning techniques are combined. Firstly, the dataset is classified by AlexNet and ResNet-18 models according to the transfer learning method. The images entered in the AlexNet form are resized to 227 × 227 × 3, whereas those in the ResNet-18 form are resized to 224 × 224 × 3. Secondly, the features extracted by the AlexNet and ResNet-18 convolutional layers are categorised by two SVM algorithms to classify the MRI images into four classes.

### 4.1. Dataset Description

System performance is evaluated using the brain tumour database. This dataset is compiled from Nanfang Hospital, Guangzhou, China, and Tianjin Medical University General Hospital, China, between years 2005 and 2010 [36]. The dataset consists of 3,060 MRI images, which are divided into four types—826 images of glioma, 937 images of meningioma, 396 images of no_tumour, and 901 images of pituitary tumour. All MRI images have the size of 512 × 512 pixels.  Figure 2 shows the MRI images of the three types of brain tumours in addition to the normal fourth type.

### 4.2. Image Enhancement

The artifacts produced by the magnetic field, normal noise, and patient movement during MRI are the challenges in analysing the MRI images of brain tumours [37]. Noise corrupts the fine detail in MRI images, reduces the spatial resolution of images, and blurs the edges of tumours [38]. Consequently, noise degrades the performance of CNN models due to complications in feature extraction [39]. For these reasons, techniques to reduce noise and contrast have been of benefit to enhance image quality. Given that MRI images are obtained from various sources, a contrast is observed in the MRI intensity from a machine computerised tomography scan to another. Therefore, intensity normalisation is applied using min–max normalisation methods to reduce the severity of homogeneity. In this work, the MRI images are enhanced through mean calculation for three RGB colour channels. Then, the images are scaled for colour constancy. Next, the input MRI images are resized. Finally, the average filter is applied for enhancing MRI. The images pass through two filters—the average filter to show the contrast and the removal of noise and a Laplacian filter to show the edges of the brain tumours. Firstly, a 4∗4 averaging filter is applied and moved around the entire image where each central pixel is replaced by the average of 15 pixels adjacent to each central pixel. Equation (1) describes the mechanism of the action of the mean filter [40].

(1) $$\begin{array}{c} z\left(m\right)=\frac{1}{M}\overset{M-1}{\underset{i=0}{\sum }}y\left(m-1\right), \end{array}$$

where *z*(*m*) is the input, *y*(*m* − 1) is the previous input, and *M* represents the number of pixels in each image.

Secondly, the images pass through the Laplacian filter to detect the edges of brain tumours with high accuracy. Equation (2) describes how the Laplacian filter works.

(2) $$\begin{array}{c} \nabla^{2}\;f=\frac{\partial^{2}\;f}{\partial^{2}\;x}+\frac{\partial^{2}\;f}{\partial^{2}\;y}, \end{array}$$

where ∇^2^ *f* is a differential equation of second order; *x*, *y* are the coordinates of the binary matrix.

Finally, the image produced by the Laplacian filter is subtracted from the image produced by the averaging filter to obtain an improved image, as presented in

(3) $$\begin{array}{c} \text{Enhanced image}=z\left(m\right)-\nabla^{2}\;f. \end{array}$$

Figure 3 describes a set of image samples of the brain tumour dataset after undergoing the enhancement process.

### 4.3. Feature Extraction

After the data augmentation process, a large dataset is trained. Features that represent each tumour are then extracted. The benefit of deep learning determines how to extract features from a training set through convolutional filters. In this study, the dataset is evaluated on AlexNet and ResNet-18 models to classify three types of brain tumours in addition to characterising normal brain images. Models contain the three most important layers: convolutional, pooling, and fully connected layers. Convolutional layers are based on the three most important parameters: filter size, padding, and pitch. Each layer contains many filters that are used to extract deep features. The filter moves in the images according to the stride. The size of the stride is one or two; if the value exceeds two, then the performance of CNNs deteriorates. When the filter in convolutional layers does not cover all the input images, zero padding is required to preserve the spatial measurements. Each convolutional layer focuses on performing a specific task; for example, the first layer highlights lesion edges, the second layer extracts complex geometric features, and the third layer highlights lesion colours and shapes. The RLU layer in a feature map passes positive values, suppresses negative values, and converts them to zero. Then, pooling layers reduce the dimensions of the extracted features. The two popular techniques in pooling layers are the average and max. Batch normalisation layers are applied to normalise feature maps. These layers speed up training and regulate the network. In this study, we extract features from the MRI images of brain tumours by the AlexNet and ResNet-18 of CNNs for feature extraction. A total of 9,216 features are derived from the latest convolutional layer and are stored in 1D vector for each image.

### 4.4. Classification Methods

#### 4.4.1. Deep Learning Models

*(1) AlexNet CNN*. Alex Krizhevsky designed the AlexNet model in 2012. The AlexNet architecture consists of 25 layers, namely, five convolutional layers for deep feature extraction; three max-pooling layers to reduce feature dimensions; two dropout layers to reduce overfitting, which works to stop 50% of neurons in each iteration but doubles the training time; three fully connected layers to diagnose input images; one SoftMax layer, which produces four classes of brain tumours; two layers of cross channel normalisation; and several ReLU layers that work after each convolutional layer to convert the negative numbers in the activation map to zero, as displayed in Figure 4. AlexNet has over six million trainable parameters [41].

*(2) ResNet-18 CNN*. Several ResNet architectures, which are based on deep architectures and different layers, such as 18, 34, 50, 101, and 152, have been developed and have demonstrated superior behaviour and precision. The Resnet-18 architecture consists of five convolutional layers to extract deep features; one average pooling layer to reduce feature dimensions; a fully connected layer; and a SoftMax layer, which produces four classes, as shown in Figure 5. The ResNet-18 architecture contains over 11.5 million parameters.  Table 1 shows the details of the layers in ResNet-18.

#### 4.4.2. Machine Learning (SVM)

Boser et al. (1992) and Vapnik (1995) developed the SVM algorithm by maximising margin and minimising risk. SVM belongs to supervised learning algorithms. Its goal is to generate decision lines or boundaries to separate datasets. These lines are called hyperplanes. The best decision limits are with the greatest margin. The algorithm works with linear and nonlinear data. Linear SVM works with separable data, as a hyperplane separates a dataset into two classes. All data points above the hyperplane belong to Class 1, data points under the hyperplane belong to Class 2, and data points within the margin close to the hyperplane are called support vectors. Margin is the distance from the hyperplane to support vectors. The algorithm separates multiclass data according to the one-for-all principle, and the process continues until the dataset is separated into several classes, {*x*_*i*_*i* = 1, 2, ⋯⋯*N*}, where *N* is the number of classes. Nonlinear SVM works with nonseparable data, as the data are converted from the original coordinate space to a new separable coordinate space *x* = *Φ* (*x*).

#### 4.4.3. Hybrid Deep and Machine Learning Techniques

In this section, we use hybrid deep and machine learning techniques to diagnose brain tumours with high efficiency. Given the computational cost, time, and hardware resources that deep learning models require to train datasets, these hybrid techniques solve these challenges. Such techniques promote the rapid implementation and solution of computational problems, require medium resources, and are inexpensive. They also contain two blocks. The first one is the CNN models that extract deep feature maps, specifically 9,216 features for each image. The second block is an SVM machine learning technique that quickly and efficiently classifies 3,060 × 9,216 deep feature maps. The dataset is divided into 80% for training and validation and 20% for testing. Figures 6(a) and 6(b) describe the hybrid techniques between CNN models and the SVM algorithm called the AlexNet+SVM and ResNet-18+SVM for classifying the brain tumour dataset.

## 5. Experimental Result

### 5.1. Splitting Dataset

The dataset comprised 3,060 MRI images divided into four unbalanced classes of which three were brain tumours and one was a normal brain image. Each class contained 826 (27%), 937 (30.6%), 901 (29.4%), and 396 (13%) images of glioma, meningioma, pituitary tumour, and no_tumour, respectively. The unbalanced dataset was processed during the training phase. It was then divided into 80% for training (2,448 images) and 20% for testing (612 images).  Table 2 describes the splitting of the dataset before and after data augmentation to balance it. The dataset must be balanced during the training phase, but not necessarily during the testing phase.  Table 2 shows that each class applied augmentation with a number of times that differs from the other classes to find a balanced dataset. The glioma class artificially increased by six times for each image, whereas the meningioma and pituitary classes increased by five times for each image. Finally, each image in the no_tumour class was generated 11 times.

### 5.2. Augmentation Technique

Data augmentation methods are helpful in balancing and increasing datasets on classes when the system is applied to a few and unbalanced datasets. This technique can be used for balancing the number of images among the MRI classes of brain tumours and for increasing the images. Augmentation techniques, such as rotation, cutting, height changing, width, filling operation, zooming, and horizontal rotation brightening, have been applied to increase images and balance classes. Considering that our dataset is unbalanced, this technique is applied, and the number of artificial images is increased for each class, unlike other classes. For example, in Class 1 (glioma), each image is increased six times. In Classes 2 and 3 (meningioma and pituitary), each image is increased five times, whereas in Class 4 (no_tumour), each image is increased 11 times to find balance and make the classes contain balanced images during the training phase, as explained in Table 2.  Figure 7 describes a set of image samples for the brain tumour dataset after applying data augmentation.

### 5.3. Training the MRI Dataset by Using CNN Models

Deep learning techniques require many images in a dataset to obtain promising accuracy. However, obtaining a huge dataset of medical images is difficult. To solve this problem, the use of pretrained deep learning model attributes on a dataset of over a million images, such as ImageNet, has been proven useful in solving new classification problems by transfer learning. The main idea of transfer learning is that deep convolutional models learn large datasets and transfer their training ability to classify new images, rather than train from scratch. The pretrained models are proven to perform better than the trained models from scratch for classifying medical images. In this study, AlexNet and ResNet-18 models based on transfer learning techniques were used to diagnose brain tumour datasets.  Table 3 shows the processes for tuning CNN models in terms of the Adam optimiser, the learning rate of 0.0001, the small-batch size for each model, maximum ageing for each model, validation frequency and training time for the two models.  Figure 8 describes the training of the ResNet-18 model and shows the training and loss process. The parameters of the two models, such as frequency, repetition per period, maximum repetition during the training phase, and implementation environment, are adjusted.

### 5.4. Evaluation Measure

Before moving on to viewing the classifier performance on the MRI image dataset of brain tumours, the weights and parameters for the AlexNet and ResNet-18 deep learning models are set in Table 3. In this study, four brain tumour MRI experiments were conducted to evaluate first the performance of CNN deep learning models AlexNet and ResNet-18 and then that of hybrid deep and machine learning techniques, AlexNet+SVM and ResNet-18+SVM. All experiments were evaluated using the accuracy, sensitivity, and specificity scale described in Equations (4), (5), and (6), respectively. Here, TP and TN are the numbers of correctly classified samples, whereas FP and FN are the numbers of incorrectly classified samples.

(4) $$\begin{array}{c} \text{Accuracy}=\frac{\text{TP}+\text{TN}}{\text{TP}+\text{TN}+\text{FP}+\text{FN}}*100\%, \end{array}$$

(5) $$\begin{array}{c} \text{Sensitivity}=\frac{\text{TP}}{\text{TP}+\text{FN}}*100\%, \end{array}$$

(6) $$\begin{array}{c} \text{Specificity}=\frac{\text{TN}}{\text{TN}+\text{FP}}*100\%. \end{array}$$

TP is the number of correctly classified (tumour) positive samples.

TN refers to the number of negative (benign) samples classified correctly.

FP is the number of benign cases classified as malignant.

FN refers to the number of malignant cases classified as benign.

### 5.5. Results of the CNN Models

The unbalanced dataset was addressed, and the overfitting problem was overcome through data augmentation. Depth feature maps were extracted for each image in the convolution layers, and the dimensions of each image were reduced in the pooling layers. Finally, deep feature maps were evaluated by fully connected layers for AlexNet and ResNet-18 models to diagnose the MRI images of brain tumours. The two models reached superior results for diagnosing brain tumours in four classes.  Figure 9(a) illustrates the confusion matrix for the AlexNet model, which reached 93.3% accuracy, 93% sensitivity, and 97.50% specificity. The AlexNet model was able to diagnose glioma with 93.3% accuracy, meningioma with 89.9% accuracy, no_tumour with 91.1% accuracy, and pituitary tumour with 97.8% accuracy.  Figure 9(b) shows the confusion matrix for the ResNet-18 model, which reached 93.8% accuracy, 93.75% sensitivity, and 97.5% specificity. The ResNet-18 model diagnosed glioma with 96% accuracy, meningioma with 87.50% accuracy, no_tumour with 92.4% accuracy, and pituitary tumour with 98.50% accuracy.

### 5.6. Results of the Hybrid CNN Models with SVM

In this section, two AI techniques, namely, deep and machine learning, were applied to extract deep feature maps and to classify the features extracted using the deep learning technique, respectively. Given that deep learning models require high specification computers, time-consuming training, and complex computational operations in classification layers (fully connected layers) with deep learning models, we classified the features extracted from deep learning by using SVM, which involves two experiments: AlexNet+SVM and ResNet-18+SVM.  Figure 10(a) describes the confusion matrix of the AlexNet+SVM model, which reached 95.1% accuracy, 95.25% sensitivity, and 98.50% specificity. The AlexNet+SVM model was able to diagnose glioma with 93.9% accuracy, meningioma with 93.6% accuracy, no_tumour with 94.9% accuracy, and pituitary adenoma with 97.8% accuracy.  Figure 10(b) shows the confusion matrix of the ResNet-18+SVM model, which attained 91.20% accuracy, 91.50% sensitivity, and 97% specificity. The ResNet-18+SVM model diagnosed glioma with 91.50% accuracy, meningioma with 86.10% accuracy, no_tumour with 92.40% accuracy, and pituitary adenoma with 95.60% accuracy.

## 6. Discussion and Comparative Study

In this research, the MRI images of a brain tumour dataset were diagnosed using two CNN models: AlexNet and ResNet-18. The same dataset was also diagnosed using hybrid techniques involving deep and machine learning, where the two deep learning models (AlexNet and ResNet-18) extracted deep feature maps and fed these features to the machine learning algorithm (SVM) to diagnose them. The confusion matrix contained correctly classified images called TP and TN and incorrectly classified images called FP and FN. Accuracy, sensitivity, and specificity were computed based on Equations (1), (2), and (3), respectively. The models obtained promising results for accuracy, sensitivity, and specificity measures. Before feeding the dataset to the models, noise and artifacts were removed with the same two filters average and Laplacian. We used the hybrid technique for many reasons, the most important of which is to achieve promising diagnostic accuracy compared to CNN models. It has a low computational cost and is fast in training the dataset. It requires low-cost computer resources compared to CNN models.

Table 4 shows the performance of all deep learning and hybrid models. The systems reached 93.30%, 94.27%, 95.10%, and 91.20% accuracy; 93%, 98.25%, 94%, and 91.50% sensitivity; and 97.50%, 98%, 98.50%, and 97% specificity for AlexNet, ResNet-18, AlexNet+SVM, and ResNet-18+SVM, respectively. AlexNet+SVM exhibited the best performance among the four experiments when using the AlexNet+SVM hybrid model. The system obtained 95.1% accuracy, 95.25% sensitivity, and 98.50% specificity.

Figure 11 describes the performance presentation of the proposed systems for the early diagnosis of the brain tumour dataset.

Figure 9(a) shows the confusion matrix of the AlexNet model, where it is noted that the model classified a glioma with an accuracy of 93.3%, where 154 out of 165 images were correctly classified while 11 out of 165 were incorrectly classified. At the same time, the model reached an accuracy of 89.8% for diagnosing meningioma, where 168 images out of 187 were classified correctly, while 19 images were classified out of 187 incorrectly. As for the pituitary tumour, the model achieved an accuracy of 97.8% in its diagnosis, as 176 images out of 180 were classified correctly, while four images were classified out of 180 incorrectly.  Figure 9(a) shows the confusion matrix of the ResNet-18 model, where it is noted that the model classified a glioma with an accuracy of 93.3%, where 154 out of 165 images were correctly classified while 14 out of 165 were incorrectly classified. At the same time, the model reached an accuracy of 93.6% for diagnosing meningioma, where 175 images out of 187 were classified correctly, while 12 images were classified out of 187 incorrectly. As for the pituitary tumour, the model achieved an accuracy of 97.2% in its diagnosis, as 175 images out of 180 were classified correctly, while 5 images were classified out of 180 incorrectly.

Figure 10(a) shows the confusion matrix of the AlexNet+SVM hybrid model, where it is noted that the model classified a glioma with an accuracy of 93.9%, where 155 out of 165 images were correctly classified while 10 out of 165 were incorrectly classified. At the same time, the model reached an accuracy of 93.6% for diagnosing meningioma, where 175 images out of 187 were classified correctly, while 12 images were classified out of 187 incorrectly. As for the pituitary tumour, the model achieved an accuracy of 97.8% in its diagnosis, as 176 images out of 180 were classified correctly, while four images were classified out of 180 incorrectly.  Figure 10(b) shows the confusion matrix of the ResNet-18+SVM hybrid model, where it is noted that the model classified a glioma with an accuracy of 91.5%, where 151 out of 165 images were correctly classified while 14 out of 165 were incorrectly classified. At the same time, the model reached an accuracy of 86.1% for diagnosing meningioma, where 161 images out of 187 were classified correctly, while 26 images were classified out of 187 incorrectly. As for the pituitary tumour, the model achieved an accuracy of 95.6% in its diagnosis, as 172 images out of 180 were classified correctly, while 8 images were classified out of 180 incorrectly.

Table 5 shows the diagnostic accuracy of the four systems for diagnosing each tumour class. The best diagnostic accuracy of glioma obtained using the AlexNet+SVM hybrid model is 93.9%, and that for meningioma achieved using the same model is 93.60%. The best diagnostic accuracy of the nontumour images attained using the AlexNet+SVM hybrid model is 94.90%. The best diagnostic accuracy of the pituitary tumour obtained using the AlexNet+SVM hybrid model is 97.8%.  Figure 12 displays the diagnostic accuracy of each class for the MRI dataset using the four models.

Table 6 and Figure 13 illustrate the performance of the proposed systems, which were evaluated using several methods in the literature survey. Several related works were also evaluated. Accuracy in previous studies ranged from 94.53% to 85%, whereas that in our system was 95.10%. Sensitivity in previous research ranged between 92.38% and 84.38%, whereas that in our system was 95.25%. Specificity in previous studies was between 95.79% and 79%, whereas that in our system was 98.50%.

## 7. Conclusion

The detection of a brain tumour is a major challenge due to the complex brain structure. The brain is responsible for controlling the functions of all the body organs. The automatic classification of early-stage brain tumours using deep and machine learning techniques plays an important role. These systems allow for timely diagnosis and increase patients' chance of survival. These techniques also help experts and radiologists in making decisions regarding diagnosis and treatment plans. We conducted four experiments to diagnose three types of MRI images of brain tumours (meningioma, glioma, and pituitary) and one class that contains healthy images. We used a new approach where we hybrid deep learning models with machine learning techniques (i.e., AlexNet, AlexNet+SVM, ResNet-18, and ResNet-18+SVM). Images were improved with the average and Laplacian filters. The enhanced images were introduced into deep learning models to extract deep and discriminatory features. Deep features were diagnosed using CNN classifiers, which are SoftMax, and machine learning classifiers called SVM algorithms. All the proposed systems yielded promising results for diagnosing MRI images of brain tumours, with little difference in accuracy among models. There are significant differences in the computational cost during training the dataset. The training of the dataset by the AlexNet model consumed 47 min 35 sec. In contrast, the computational cost of training the dataset by the ResNet-18 model was 349 min 13 sec. It is noted that the computational cost is high. In contrast, when applying the hybrid techniques between CNN models and the SVM algorithm, the computational cost was low as follows. The dataset was trained by the AlexNet+SVM hybrid model through 3 min 21 sec, while the computational cost of training the dataset by the ResNet-18+SVM hybrid model was 2 min 23 sec. A laptop Intel ® i5 laptop 6 generations, 12 GB RAM, and 4 GB GPU GEFORCE, is used to run the experiments. The AlexNet+SVM hybrid model exhibited the best performance among others. Specifically, it achieved 95.1%, 95.25%, and 98.50% accuracy, sensitivity, and specificity, respectively.

## Figures and Tables

**Figure 1:** General structure of the combination of deep and machine learning techniques.

**Figure 2:** Samples of a dataset of an MRI of brain tumours. Source: (https://www.kaggle.com/sartajbhuvaji/brain-tumor-classification-mri).

**Figure 3:** Samples of the dataset after the enhancement process.

**Figure 4:** AlexNet architecture.

**Figure 5:** ResNet-18 architecture.

**Figure 6:** Hybrid architecture between deep and machine learning: (a) AlexNet+SVM; (b) ResNet-18+SVM.

**Figure 7:** A set of image samples after applying data augmentation.

**Figure 8:** Training and loss process of the ResNet-18 model.

**Figure 9:** (a) Confusion matrix for AlexNet to evaluate MRI brain tumours. (b) Confusion matrix for ResNet-18 to evaluate MRI brain tumours.

**Figure 10:** (a) Confusion matrix for AlexNet+SVM to evaluate MRI brain tumours. (b) Confusion matrix for ResNet-18+SVM to evaluate MRI brain tumours.

**Figure 11:** Performance of the proposed systems for the brain tumour dataset.

**Figure 12:** Performance of the four models for the detection of each brain tumour.

**Figure 13:** Performance comparison of the proposed systems with related studies.

**Table 1:** Detailed structure of the ResNet-18 CNN.

Layer	Conv 1	Conv2.x		Conv3.x		Conv4.x		Conv5.x		Pooling
Output size	112 × 112 × 64	56 × 56 × 64		28 × 28 × 128		14 × 14 × 256		7 × 7 × 512		1 × 1 × 512
Filter	7 × 7, 64 stride 2	3 × 3, 64	×2	3 × 3, 128	×2	3 × 3, 256	×2	3 × 3, 512	×2	Average
		3 × 3, 64		3 × 3, 128		3 × 3, 256		3 × 3, 512		

**Table 2:** Balancing the MRI images of the brain tumour dataset during the training phase.

Phase	Training phase 80%			
Class name	Glioma	Meningioma	Pituitary	No_tumour
No images before augmentation	661	750	720	317
No images after augmentation	3,965	3,750	3,600	3,487

**Table 3:** Adjusted training parameters of ResNet-18 and AlexNet models.

Option	AlexNet	ResNet-18
Training option	Adam	Adam
Minimum batch size	135	15
Maximum epoch	10	8
Initial learn rate	0.0001	0.0001
Validation frequency	50	5
Training time (min)	47 min 35 sec	349 min 13 sec
Execution environment	GPU	GPU

**Table 4:** Results of diagnosing brain tumours using deep learning models and hybrid deep and machine learning techniques.

Classifier	Deep learning		Hybrid deep and machine learning techniques	
	AlexNet	ResNet-18	AlexNet+SVM	ResNet-18+SVM
Accuracy (%)	93.3	93.8	95.1	91.2
Sensitivity (%)	93	93.75	95.25	91.5
Specificity (%)	97.5	97.5	98.5	97

**Table 5:** Diagnostic accuracy of the four models for diagnosing each tumour class.

Tumour type	AlexNet	ResNet-18	AlexNet+SVM	ResNet-18+SVM
Glioma	93.30	93.3	93.90	91.50
Meningioma	89.80	93.6	93.60	86.10
No_tumour	91.10	87.3	94.90	92.40
Pituitary	97.80	97.2	97.80	95.60

**Table 6:** Comparing the performance of the proposed systems with relevant studies.

Previous research	Accuracy (%)	Sensitivity (%)	Specificity (%)
Sharif et al. [18]	92.5	—	—
Dandu et al. [19]	90.2	—	—
Amin et al. [20]	87	92	80
Huang et al. [21]	94.53	—	—
Kaur et al. [22]	91.51	90.65	95.79
Kumar et al. [24]	92.63	92.38	93.33
Afshar et al. [42]	92.45	90.36	91.98
Bahadure et al. [43]	92.03	92.36	91.42
Toğaçar et al. [44]	87.93	84.38	92.31
Zollner et al. [45]	85	89	84
Amarapur [46]	89	85	91
Cho et al. [47]	89.81	88.89	90.74
Ghassemi et al. [48]	91.7	90.16	95.58
David et al. [49]	85	87	79
*Proposed model*	**95.1**	**95.25**	**98.5**

## Data Availability

The datasets were collected from Nanfang Hospital, Guangzhou, China, and Tianjin Medical University General Hospital, China, between years 2005 and 2010. Available at this link: https://www.kaggle.com/sartajbhuvaji/brain-tumor-classification-mri.
